The article "Role of Livelihood Capital in Reducing Climatic Vulnerability: Insights of Australian Wheat from 1990–2010" was retracted in 2022. Reason: duplicate publication.

# Role of Livelihood Capital in Reducing Climatic Vulnerability: Insights of Australian Wheat from 1990–2010

**DOI:** 10.1371/journal.pone.0152277

**Published:** 2016-03-29

**Authors:** Jianjun Huai

**Affiliations:** Department of Economics, College of Economics and Management, Northwest A&F University, Yangling, Shaanxi, China; Murdoch University, AUSTRALIA

## Abstract

In many agricultural countries, development of rural livelihood through increasing capital is a major regional policy to adapt to climate change. However, the role of livelihood capital in reducing climatic vulnerability is uncertain. This study assesses vulnerability and identifies the effects of common capital indicators on it, using Australian wheat as an example. We calculate exposure (a climate index) and sensitivity (a wheat failure index) to measure vulnerability and classify the resilient and sensitive cases, and express adaptive capacity through financial, human, natural, physical, and social capital indicators for 12 regions in the Australian wheat–sheep production zone from 1991–2010. We identify relationships between 12 indicators of five types of capital and vulnerability with *t*-tests and six logistic models considering the capital indicator itself, its first-order lag and its square as dependent variables to test the hypothesis that a high level of each capital metric results in low vulnerability. Through differing adaptive capacities between resilient and sensitive groups, we found that only four of the 12 (e.g., the access to finance, cash income level, total crop gross revenues, and family share of farm income) relate to vulnerability, which challenges the hypothesis that increasing capital reduces vulnerability. We conclude that further empirical reexaminations are required to test the relationships between capital measures and vulnerability under the sustainable livelihood framework (SLF).

## Introduction

The adverse effects of extreme climate events have destroyed rural livelihoods because of the loss of crops in agricultural regions. In most of the world's wheat-growing areas, climate change has reduced the production of wheat [1], which threatens rural livelihoods. According to the sustainable livelihoods framework (SLF), the development of livelihood capital enhances livelihood outcomes including reduced vulnerability [2]. Thus, many regional governments encourage householders to improve their rural livelihood capital to adapt to the risk of climate change. However, the impact of this ‘increasing-capital’ method rests on the influence of livelihood capital on the vulnerability of crops to climate change.

Although many studies have reviewed the theory of vulnerability and adaptive capability to climate change [3–6], there is a general disagreement regarding the influences of adaptive capacity on crop vulnerability at various contexts and levels [7–9]. Vulnerability has a nested hierarchy relationship with adaptation, adaptive capacity, resilience, sensitivity and exposure, which leads to a complex and potentially confusing process for assessing vulnerability [7]. Different typologies of crop-drought vulnerability are associated with different adaptation measures according to their regional constraints. For example, increased agricultural investments were shown to increase the resilience of crops to drought in sensitive regions, while simultaneously increasing crop-drought vulnerability in resilient regions in China [10]. In addition, numerous critical factors without accurate measures, e.g., combined socioeconomic ecological systems, multiple climate elements, scales of time and space, components and structures of vulnerability, and uncertainties in adaptations lead to a complex influence of livelihood capital on synthesized vulnerability [8].

As one of the more robust resolutions to the above-mentioned challenges, the SLF developed by the United Kingdom Department for International Development (UK DFID) states that the improvement of livelihood capital reduces vulnerability in the processes of decision and response. Sustainable livelihood analysis includes the following steps. First, some vulnerability contexts are recognized and defined (e.g., external shocks), in which stakeholders should estimate their perceived and actual vulnerability, and adjust their current asset portfolios (including financial, human, natural, physical, and social). Second, the transforming organization structures and the operating processes of institutions, cultures, laws, and policies affect the asset portfolios and choice of the livelihood strategies at multiple levels, and react to the vulnerability context. Third, proposed livelihood outcomes (increased well-being and income, improved food security, reduced vulnerability, and sustainable use of natural resources) are achieved step by step, which also changes the portfolios of livelihood assets [2]. The SLF emphasizes the population’s social and economic activities, assesses inter-sector management and intervention, and is also responsive and participatory, strengthens stakeholder capabilities, and takes a broad and dynamic approach to sustainability [11]. Many methods of increasing capital, (such as rising access to diverse livelihood resources, growing efficiency of portfolio management of assets, and promoting socioeconomic development), enhance rural livelihoods and adaptive capacity, and decrease vulnerability to climate change [12, 13]. Therefore, ‘increasing capital’ is considered to constitute a good method to reduce vulnerability [14, 15].

However, the role of livelihood capital opposes the ‘increasing capital’ method for reducing vulnerability. Many advancing livelihood capitals do not reduce vulnerability until after the point in which community resilience is developed [16]. Some scholars simply assume that livelihood capital complements the adaptive policy [17]. Furthermore, the increase of livelihood capital has led stakeholders into unsustainable livelihoods in some regions [18]. Some livelihood capital indicators can reduce vulnerability while others can simultaneously increase it. For example, high infrastructure index (physical capital) and high literacy rates (human capital) reduce vulnerability, while high shares of agriculture in total GDP (financial capital), densely populated rural areas (physical capital), high dependency on rain-fed agriculture, and high land degradation (natural capital) increase it [19]. A strong bonding network could perpetuate and exacerbate, rather than reduce, vulnerability, and social capital has a complex, but uniformly positive, relationship with climatic vulnerability [20]. The complementary interactions and substitutions of each capital indicator are too complex to measure, and thus indicators are assumed to complement each other simply, which obscures the individual impact of each indicator on the vulnerability [21]. Such conflicts between theories challenge the increasing-capital method.

The purpose of this study is to estimate vulnerability, identify resilient and sensitive cases, and detect the role of livelihood capital on reducing vulnerability. In this study, we quantified the wheat vulnerability to climate change at 12 regions in the Australian wheat—sheep production zone during 1991–2010 to determine whether livelihood capital reduces climatic vulnerability. Driven by the IPCC-SLF, we hypothesized that some elements of livelihood capital influence exposure and sensitivity, confer adaptive capacity, and significantly reduce wheat climatic vulnerability. Vulnerability is composed of exposure (climate index measured by average maximum temperature on the crop shelf) and sensitivity (wheat failure index calculated from wheat yields contributed in surveys). The vulnerability of wheat to climate change (calculated by the ratio of the wheat failure index to the climate index) was ranked by quartiles to identify sensitive and resilient cases. We determine relationships between 12 indicators of five forms of capital (financial, human, natural, physical, and social) and vulnerability with Student’s *t*-tests and a logistic regression to test the hypothesis that high levels of each capital metric result in low vulnerability. We illustrate the classification of vulnerability at different spatial and temporal levels, and assess the influence of capital metrics on vulnerability. We then discuss the different methods for assessing vulnerability, the mechanism through which the significant capital indicators affect vulnerability, and the reasons for the low number of capital indicators affecting vulnerability.

## Methods

### Study area: Australian wheat—sheep production zone

As having the world's fifth-highest per capita income in 2014 and one of the most important wheat growing countries, Australia has rich livelihood capital, including a high-quality of life, health, advanced education, and economic freedom. As the second largest wheat exporter in the world, Australia exports wheat to about 40 countries, and is highly competitive in international food markets. However, the rising trend in temperatures and the chronic shortages of water because urban population increases and localized drought have led to doubt regarding the sustainability of these livelihoods. For example, the sustainability is influenced in 2030, profitability in 2050 and biodiversity in 2070 by increasing drought and decreasing precipitation in Western Australia [22]. Therefore, it is emergent for Australian governments to assess the vulnerability of crops to climate change and the role of ‘building-capital’ methods to reduce such vulnerability.

Wheat is the highest value crop with the largest planting area in Australia. Ninety percent of wheat is produced in the Australian wheat—sheep production zone designated by the Australia Bureau of Agricultural and Resource Economics and Sciences (ABARES). The overall area of this zone, composed of 12 regions, is 109.728 million ha, with around 11 billion hm^2^ of wheat planting area and 22 billion tons of average production per year. In these areas, the precipitation is 170–400 mm during the wheat-growing season, and less than 4% of the area is irrigated. In recent decades, the climate has become drier and more drought-prone, and the increased temperatures and decreased rainfall has severely affected the wheat crop. For example, the 2007 drought caused wheat production to fall by about 60% in the wheat—sheep production zone [23]. In the future, higher temperatures and less rainfall are likely to reduce wheat yield, further increase wheat vulnerability, and threaten farmers’ livelihoods [24, 25].

This context and the good availability of data make the Australian wheat—sheep production zone a suitable study area to evaluate the relationship between livelihood capital and the vulnerability of wheat to climate change.

### Assessing wheat climatic vulnerability and livelihood capital

We tested the role of livelihood capital in the reduction of wheat climatic vulnerability using the following steps. First, we structured the vulnerability into elements of exposure, sensitivity and adaptive capacity, and selected proxy indicators from the Australian Agricultural and Grazing Industries Survey (AAGIS). According to the definition of livelihood capital and previous studies [26–28], we selected available annual indicators from AAGIS (1990–2010) as proxies of financial, human, natural, physical, and social capital in the wheat—sheep production zone. Because of the variable availability and quality of data, we had to accept some limitations to the study. For example, there were only two or three indicators to present human capital because educations data were not available to the study (Table 1). Second, we identified years with considerable climate variation as the exposure indicator, using a climate index, wheat yield abnormal years as sensitivity using a wheat failure index, and adaptive capacity using elements of financial, human, natural, physical, and social capital. We classified resilient and sensitive groups by defining the first quartile and the fourth quartile of the vulnerability index. Third, assuming that sensitive groups have higher vulnerability and lower adaptive capacity than resilient ones, we hypothesized that each selected indicator of the five capitals is negative with the probability of vulnerability for sensitive groups. Finally, we applied Student’s *t*-test and a logistic model for two independent samples (resilient and sensitive cases) to identify influential capital elements of wheat climatic vulnerability.

**Table 1:** Definitionof Capital Indicators.

Capital Indicator	Definition
Total crop gross revenues (TCGR_NC) a	Total gross revenues from sale of crops and hay during the survey year.
Effective rainfall on the crop (ER_NC) b	Effective rainfall on the crop in the planting areas.
Fertilizer expenditure (FE_NC) a	Expenditure on fertilizers and soil conditioners during the survey year.
Electricity expenditure (EE_PC)^a^	Expenditure on electricity.
Land value and improvements (VLI_PC) a	Market value of all land operated and fixed improvements starting at the end of the financial year estimated by the owner-manager or co-operator.
Age of owner manager (AOM_HC) a	Age of the primary decision-maker in the farm business.
Total labor use (TLU_HC) a	Total number of full time weeks worked by all farm workers, including hired labor.
Average cash income level (ACIL_FC)^a^	Average cash income level in the nth year is the average of cash income in the previous n−1 years, where n equals 1, 2…20 for each region.
Access to finance (AF_FC) a	Access to finance equals borrowing capacity plus liquid assets. Borrowing capacity is derived from each farm’s equity ratio. When the equity ratio is less than 70 percent, borrowing capacity is zero; otherwise, borrowing capacity = (equity ratio − 0.70) × capital (see TCC_FC).
Total closing capital(TCC_FC) a	Closing value of all assets used on the farm including leased equipment, but excluding machinery and equipment either hired or used by contractors.
Family share of farm income (FSFI_SC) a	Ownership share of total cash income of owner-manager, spouse, and dependent children.
Telephone charges (TC_SC) a	Telephone charge.

Notes: FC, Financial capital; HC, Human capital; NC, Natural capital; PC, Physical capital; SC, Social capital; 1$K, $1000; 1$M, $1,000,000;

The survey years range from 1990 to 2010.

^a^. Data Recourse: https://apps.daff.gov.au/AGSURF/.

^b^. Data Recourse: Bureau of Meteorology.

Reference: [14, 27, 28].

### Assessment of wheat climatic vulnerability

Vulnerability is composed of exposure (the degree of significant variation), sensitivity (the response to the variation), and adaptive capacity (the ability to adapt to the variation)[29]. Here, maximum annual temperature represent the exposure of climate change, actual wheat yields represent the sensitivity of crops to climate change.

We calculated the climate index (CI) as a ratio of the maximum annual temperature on the crop shelf for region *r* and year *i* to the mean annual maximum temperature for each region over all years minus one, as follows:

$$CI_{ri}=\frac{T_{\text{ri}}}{\bar{T_{\text{r}}}}-1$$ (1)

The measure of sensitivity, which reflects the response of wheat to climate change, was calculated such that the wheat failure index (WFI) is the regional average wheat yield of overall years divided by(survey—reported) actual wheat yield selected from AAGIS from 1991–2010 for region *r* and year *i* minus one, as follows:

$$WFI_{ri}=\frac{\bar{Y_{r}}}{Y_{ri}}-1$$ (2)

We can assess the wheat climatic vulnerability in Australia according to the measurements of exposure and sensitivity of wheat to climate change. Similarly to [10], comparing *CI* and *WFI*, we assessed the wheat climatic vulnerability index (VI) in each region and year using Eq (3):

$$WVI_{ri}=\frac{WFI_{\text{ri}}}{CI_{\text{ri}}}$$ (3)

#### Classifying resilient and sensitive groups

Wheat cultivated in diverse regions respond to the climate warming in different ways and thus some years or regions are more vulnerable than others [30, 31]. For example, the wheat yield was 18–22% lower than the normal yield in dry regions under climate warming [32]. Therefore, classifying vulnerable or climate variation years (*groups*)constitutes the focus of the present work. We then stratified the climate variation years into sensitive (S) and resilient (R) groups using the quartile method. A year is considered resilient if its vulnerability lies within the first quartile of *WVI*, where high exposure causes low sensitivity. A year is considered sensitive if its vulnerability lies within the fourth quartile of *WVI*, where low exposure causes high sensitivity. Such classifications identify high vulnerability in the sensitive groups and low vulnerability in the resilient groups (Table 2). Furthermore, we identify the resilient regions from sensitive regions according to the lines of *WVI* from 1990–2010.

**Table 2:** Descriptions of dependent variables.

	N	Min	Max	Mean	St.D
CRL_NC	118	3.57E+04	8.99E+05	2.16E+05	1.56E+05
ER_NC	118	2.19E+01	2.70E+02	1.48E+02	4.89E+01
FE_NC	118	1.85E+03	1.45E+05	3.52E+04	3.28E+04
EE_PC	118	1.08E+03	6.12E+03	2.58E+03	9.67E+02
VLI_PC	118	6.62E+05	5.03E+06	1.87E+06	9.47E+05
AOM_HC	118	4.30E+01	6.00E+01	5.34E+01	3.04E+00
TLU_HC	118	7.80E+01	1.51E+02	1.05E+02	1.39E+01
ACIL_FC	111	4.16E+04	1.84E+05	9.90E+04	3.18E+04
AF_FC	108	5.94E+07	4.86E+08	1.84E+08	8.65E+07
TCC_FC	118	8.26E+05	6.13E+06	2.32E+06	1.15E+06
FSFI_SC	118	−1.01E+05	2.09E+05	1.02E+04	3.87E+04
TC_SC	118	1.18E+03	6.13E+03	2.44E+03	8.58E+02
CRL_NC(−1)	111	3.57E+04	6.84E+05	2.23E+05	1.47E+05
ER_NC(−1)	111	4.52E+01	2.66E+02	1.51E+02	5.07E+01
FE_NC(−1)	106	1.85E+03	1.45E+05	3.40E+04	3.15E+04
EE_PC(−1)	111	1.02E+03	6.12E+03	2.57E+03	9.43E+02
VLI_PC(−1)	111	6.62E+05	4.93E+06	1.82E+06	8.93E+05
TLU_HC(−1)	111	7.70E+01	1.51E+02	1.06E+02	1.46E+01
ACIL_FC(−1)	105	3.70E+04	1.89E+05	9.74E+04	3.28E+04
AF_FC(−1)	103	7.13E+07	4.83E+08	1.80E+08	8.24E+07
TCC_FC(−1)	111	8.26E+05	6.09E+06	2.26E+06	1.09E+06
FSFI_SC(−1)	111	−1.01E+05	1.16E+05	1.62E+04	3.54E+04
TC_SC(−1)	111	1.19E+03	6.13E+03	2.47E+03	8.94E+02
CRL_NC_S	118	1.27E+09	8.08E+11	7.06E+10	1.19E+11
ER_NC_S	118	4.79E+02	7.28E+04	2.44E+04	1.49E+04
FE_NC_S	118	3.44E+06	2.10E+10	2.30E+09	4.52E+09
EE_PC_S	118	1.16E+06	3.74E+07	7.58E+06	5.73E+06
VLI_PC_S	118	4.38E+11	2.53E+13	4.40E+12	4.90E+12
AOM_HC_S	118	1.85E+03	3.60E+03	2.86E+03	3.21E+02
TLU_HC_S	118	6.08E+03	2.28E+04	1.13E+04	3.04E+03
ACIL_FC_S	111	1.73E+09	3.37E+10	1.08E+10	7.19E+09
AF_FC_S	108	3.53E+15	2.37E+17	4.13E+16	4.20E+16
TCC_FC_S	118	6.82E+11	3.76E+13	6.70E+12	7.17E+12
FSFI_SC_S	118	2.12E+03	4.37E+10	1.59E+09	4.46E+09
TC_SC_S	118	1.38E+06	3.76E+07	6.68E+06	5.39E+06
CI	118	−2.18E-01	2.98E-01	-4.09E-02	9.03E-02
WFI	118	−6.00E-01	2.89E+00	2.53E-01	8.22E-01
VI	118	−7.10E+01	1.12E+02	1.29E+00	2.28E+01
P(Y)	118	0.00E+00	1.00E+00	5.00E-01	5.02E-01
Number of cases	80				

**Notes**: FC, Financial capital; HC, Human capital; NC, Natural capital; PC, Physical capital; SC, Social capital; TCGR, Total crop gross revenues; ER, Effective rainfall on the crop; FE, Fertilizer expenditure; EE, Electricity expenditure; VLI, Land value and improvements; AOM, Age of owner manager; TLU, Total labor use; ACIL, Average cash income level; AF, Access to finance; TCC, Total closing capital; FSFI, Family share of farm income; TC, Telephone charges; CI, Climate index; WFI, Wheat failure index; VI, Vulnerability index; P(Y), Probability of resilient cases. (−1) and S defined the square of capital indicator, for example, TC_SC (−1) and TC_SC_S is the fist-order lag and square of TC_SC.

All data comes from S1 Dataset

### Influence of the development of livelihood capital on vulnerability

To understand the role of livelihood capital, we hypothesized that each capital indicator of livelihood (e.g., natural, physical, human, financial and social) capital reduces the drought vulnerability of wheat. We also investigated the influences of each capital indicator on the vulnerability of wheat to climate change in the wheat—sheep production zone.

Natural capital (NC) is the stock of natural resources that create a long-term supply of goods or services. Here we used total crop gross revenues, effective rainfall on the crop shelf, and fertilizer expenditures to measure NC. The total crop gross revenue comes from the sales of crops (including wheat, barley, and oats) and hay during the survey year, in which higher total crop gross revenue indicates good supply of the main crops. Rainfall influences crop production [33]. Scarce rainfall is known to ruin the harvest when the crop blooms, especially in semi-arid areas [34]. Various fertilizer managements can reduce the vulnerability of climate change through increasing the longer-term soil organic elements and also tend to increase N_2_O emissions and reduce the CH_4_ emissions [35–37]. Thus, the decline of crop revenues and effective rainfall could enhance wheat climatic vulnerability by reducing wheat yield and production, while fertilization expenditures have a nonlinear effect on climatic vulnerability.

Physical capital (PC) is a factor of production, consisting here of electricity, and land value and improvements. Poor infrastructure, obsolete technology, and low access to resources can cause high vulnerability [38]. Conversely, higher land value and improvements imply better land and advanced technology. Improved infrastructure (i.e., electricity) reduces wheat vulnerability through increasing adaptive capacity to climatic disasters [39, 40]. Electricity offers sufficient power and convenient transportation to the farming system, particularly during abnormal weather conditions. Therefore, higher electricity expenditure, and land value and improvement present better PC that can reduce vulnerability on farms. However, the impacts of off-farm electricity and improvements on the vulnerability of crops to climate change remain unclear.

Human capital (HC) refers to the farmer’s indigenous knowledge, education, age, labor skills, health and women's empowerment [41] and determines the assets and labor return for farmers [42], which increase labor productivity and land management ability. Here, HC is expressed as the manager’s age and the labor used per week on the farm. Older managers are vulnerable because they generally have low strategic skills and low interest in changing behavior, while younger managers have a stronger psychological and financial buffer [43]. For example, younger managers are likely to have less experience and special skills on farms, while older managers have accumulated amounts. However, financing can make up for deficiencies in farming experience [44]. Therefore, we hypothesize that there is a non-linear relationship between age and vulnerability on the farm. The high qualities and quantities of labor inputs on the farms add the resilience of crops (e.g., rice and maize) in extreme events [45], and thus a higher number of laborers working on the farm can reduce climatic vulnerability. Because there is no available education data in the socioeconomic indicators in AAGIS, we were unable to match the education data from other surveys with AAGIS at the same spatial and temporal scales. For this reason, we had to ignore the education variable in our study.

Indicators of financial capital (FC) include average cash income levels in the previous year, current access to credit, and total closing capitals in this study [46]. Given the natural and socio-economic conditions on farms in the short-term, rational farmers have to adjust their financial activities to adapt to climate variability and change. The farmers have considerable access to transforming their income into current agricultural investments, which adds many opportunities and alternatives to resolving issue associated with droughts and water scarcity in wheat growing periods. Access to financial, technological, and information resources constitutes one of influences of adaptive capacity, which is the basis of many financial activities [7, 47]. Improved accessibility to credit can also encourage farmer confidence, add to their borrowing and lending capacities, and speed up capital liquidity. This accessibility can protect wheat production from extreme climate events by undertaking wheat trade quickly, and facilitate farmers to enter markets and purchase technology and other resources. Total closing capital represents the closing value of all assets used on the farm including leased equipment. Higher closing capital means that more investments on the farm are available to reinforce infrastructure and water equipment to improve climate change resilience [48]. Hence, we hypothesize that FC reduces wheat climatic vulnerability.

Generally, social capital (SC) emphasizes relationships of trust, membership of groups, user associations, common rules, communal rights, participatory management, and collective actions [41]. Here, SC was evaluated by the family's share of farm income and telephone charges, and was hypothesized to reduce vulnerability. The Family share of farm income presents a type of property right that determines adaptive capacity [49] and helps farmers to better manage adverse climate events because increased family involvement reduces transformation costs. Superior communications regarding adaptations can also reduce climatic vulnerability. When farmers share information through telephone communications in agricultural networks, they collectively manage the farm, increase farm income, and thus reduce crop system vulnerability [50].

#### Testing the influence of capital metrics

Under the SLF, we selected 12 indicators of five forms of capital, and then tested whether each indicator is related to the wheat climatic vulnerability. We utilized a construct model to present the role of livelihood capital indicators in reducing wheat climatic vulnerability (Fig 1). In contrast to the common practice of simply assuming that high levels of livelihood capital can engender adaptive capacity and reduce vulnerability, we identified complex impacts of each of the five capital indicators itself, its first-order lag and its square on the vulnerability with *t*-tests and a logistic model to test the hypothesis that high levels of each capital metric result in low vulnerability.

**Fig 1:** Influences of capital indicators on the reduced vulnerability under the SLF. This constructed model ignores perceived vulnerability, assets portfolios, structures and processes, and achieved order of livelihood outcomes.

A set of *t*-tests for two independent samples, including the Levene’s tests for equality of variances, were performed to quantify differences in these indicators between resilient and sensitive groups. The null hypothesis of the *t*-test indicates that the mean of the capital indicator for the resilient groups equals its mean for sensitive groups. Levene’s test employs the null hypothesis, such that the variance of the capital indicator for resilient groups equals its variance for sensitive groups.

We also estimated a logistic model with the dummy variable for vulnerability as the dependent variable and capital indicators as the independent variables. Specifically, we estimate the following model:

$$p{\left(Y=1,0\right)}_{j}=\alpha_{0}+\sum_{i=1}^{12}\alpha_{1}x_{i}+\sum_{j=0}^{1}\sum_{i=1}^{12}\alpha_{1}x_{i}(-1)+\sum_{k=0}^{1}\sum_{i=1}^{12}\alpha_{1}x_{{}_{i}}^{2}+\mu_{i}(i=1,2,\ldots ,12;j,k=0,1)$$ (4)

where *p* is a binary dummy variable (*Y* = 1 for resilient cases, *Y* = 0 or sensitive cases), *x* stands for 12 capital indicators listed in Table 1, *x*(-1) presents the first-order lag of *x*, the *u* is an error term.

Eq (4) was estimated using a logistic model to account for the fact that the dependent variable is binary, which can illustrate the effect of each variable on the likelihood that *Y* fall into the resilient group. Eq (4) breaks down into six models that can represent a range of capital roles on the vulnerability, as shown below:

$$\text{Model 1: }p{\left(Y=1,0\right)}_{j}=\alpha_{0}+\sum_{i=1}^{12}\alpha_{i}x_{i}+u_{i}(i=1,2,\ldots 12)$$ (5)

$$\text{Model 2: }p{\left(Y=1,0\right)}_{j}=\alpha_{0}+\sum_{i=1}^{12}\alpha_{i}x_{i}(-1)+u_{i}(i=1,2,\ldots 12)$$ (6)

$$\text{Model 3: }p{\left(Y=1,0\right)}_{j}=\alpha_{0}+\sum_{i=1}^{12}\alpha_{i}x_{i}^{2}+u_{i}(i=1,2,\ldots 12)$$ (7)

$$\text{Model 4: }p{\left(Y=1,0\right)}_{j}=\alpha_{0}+\sum_{i=1}^{12}\alpha_{i}x_{i}+\sum_{i=1}^{12}\alpha_{i}x_{i}(-1)+u_{i}(i=1,2,\ldots 12)$$ (8)

$$\text{Model 5: }p{\left(Y=1,0\right)}_{j}=\alpha_{0}+\sum_{i=1}^{12}\alpha_{i}x_{i}+\sum_{i=1}^{12}\alpha_{i}x_{i}^{2}+u_{i}(i=1,2,\ldots 12)$$ (9)

$$\text{Model 6: }p{\left(Y=1,0\right)}_{j}=\alpha_{0}+\sum_{i=1}^{12}\alpha_{i}x_{i}+\sum_{i=1}^{12}\alpha_{i}x_{i}(-1)+\sum_{i=1}^{12}\alpha_{i}x_{i}^{2}+u_{i}(i=1,2,\ldots 12)$$ (10)

Each capital indicator was selected from AAGIS according to the deductive definition of every type of livelihood capital. Other data, e.g., wheat yield, was also selected from AAGIS. For the past few decades, AAGIS had an annual survey about farm’s input-output at the farmer’s level, which has been popular for use by scientists in Australia and globally. The climatic data, such as temperature, originates from the Bureau of Meteorology (BOM) and are often used to estimate the APSIM modeling.

## Results

### Data descriptions

All data have the statistical descriptions as shown in Table 2.

### Assessing wheat climatic vulnerability and classifying resilient and sensitive cases

Fig 2 shows the temporal and spatial changes of *WVI*, which provide a detailed classification of resilient and sensitive cases of wheat to climate change in Australia's wheat—sheep production zone from 1991–2010. Through comparing the curves of mean *WVI* in each region during 1991–2010, we identified the resilient and sensitive cases. For example, the sensitive cases are the years that have high vulnerability (e.g., 1995 in the Riverina), and the resilient cases are the years that have low vulnerability (e.g., 2010 in the Central and South Wheat Belt). The cases with the greatest *WVI* do not match with the cases with the lowest *WVI* in most regions. For example, the lowest *WVI* occurred in 1992 in the North and East Wheat Belt, while the lowest *WVI* occurred in 1996 in the North West Slopes and Plains.

**Fig 2:** Line graphs of wheat vulnerability to climate change (WVI) across all regions from 1991 to 2010 in the Australian wheat—sheep production zone.

We also classified the vulnerable regions by comparing the variances of *WVI* (Fig 2), because their smaller variances present few changes of vulnerability of wheat to climate change. At the state level, South Australia and Victoria exhibit the lowest variance of *WVI*, and are therefore resilient; Queensland is moderate, while West Australia and New South Wales have the highest variance and are considered as sensitive states. At the regional level, the Darling Downs and Central Highlands in QLD, Central North, and Wimmera are considered as resilient regions because these regions show no clear variances of *WVI* since 1990. Other regions with more than three sensitive cases (years) are considered to be as sensitive regions, e.g., the North and East Wheat Belt, the Central and South Wheat Belt, and Mallee.

Independent tests were performed to determine whether there were significant differences between resilient and sensitive cases for wheat in regard to their climatic vulnerability in different regions and years. Table 3 indicates that there was a significant difference between the two groups for the *CI* and *WFI* sampled, in regard to their wheat climatic vulnerability, compared to abnormal years. The sensitive cases had a 0.036 higher mean *CI* than resilient cases, reflecting a smaller abnormal climate (exposure), and a 0.535 lower mean *WFI*, indicating a greater wheat loss (sensitivity). In total, higher sensitivity followed by lower exposure causes higher vulnerability over time.

**Table 3:** Comparison of capital indicators on vulnerability in different groups.

Variables	Groups	Hypothesis	T	Sig.(Two-tailed)	Mean Difference
ER_NC	S	E	−2.208	0.029	−1.96E+01
	R	EN			
VLI_PC	S	E	−2.185	0.031	−3.75E+05
	R	EN			
ACIL_FC	S	E	−2.008	0.047	−1.20E+04
	R	EN			
AF_FC	S	E	−1.666	0.099	−2.76E+07
	R	EN			
TCC_FC	S	E	−2.204	0.030	−4.57E+05
	R	EN			
FSFI_SC	S	E	3.138	0.002	2.16E+04
	R	EN			
ER_NC(−1)	S	E	−2.45	0.016	−2.30E+01
	R	EN			
VLI_PC(−1)	S	E	−2.203	0.030	−3.67E+05
	R	EN			
ACIL_FC(−1)	S	E	−1.987	0.050	−1.25E+04
	R	EN			
AF_FC(−1)	S	E	−2.218	0.029	−3.54E+07
	R	EN			
TCC_FC(−1)	S	E	−2.364	0.020	−4.79E+05
	R	EN			
ER_NC_S	S	E	−2.179	0.031	−5.88E+03
	R	EN			
ACIL_FC_S	S	E	−1.831	0.070	−2.47E+09
	R	EN			
CI	S	E	2.232	0.028	3.65E-02
	R	EN			
WFI	S	E	−3.721	0.000	−5.35E-01
	R	EN			

Notes: p < 0.05; CI, climate change index; WFI, wheat failure index; V, vulnerability; R, resilient groups; S, sensitive groups; E, Equal variances assumed; EN, Equal variances not assumed.

### Effects of livelihood capital metrics on wheat climatic vulnerability

When considering adaptive capacity, we illustrated that there are limited statistically significant effects of livelihood capital on wheat climatic vulnerability. Table 3 indicated that there was no significant difference between two groups for the capital indicators sampled, in regard to their wheat climatic vulnerability. Table 3 shows that only 10 of the 36 indicators are significantly different between the resilient and sensitive groups at a 95% confidence level, which means that only 10 correlate with vulnerability. The resilient cases have more effective rainfall (ER_NC) (19.55 mm), land value and improvements (VLI_PC) (0.375 million dollars per year), average cash income level (ACIL_FC) (11.972 thousand dollars per year), and access to finance (AF_FC) (27.599 million dollars per year) than the sensitive cases. This suggests that higher levels of FC tended to reduce vulnerability. However, the sensitive cases have a 21.551 thousand dollars higher family share of farm income (FSFI_SC) than sensitive cases. The first-order lag variables of these four capital indicators, i.e., ER_NC (−1), VLI_PC (−1), ACIL_FC (−1) and AF_FC (−1), have impacts on vulnerability. For example, the resilient cases have a 23.04 mm higher effective rainfall (ER_NC (−1)) than the sensitive cases. In contrast, the resilient cases have a 0.479 million dollars higher first-order lag total closing capital (TCC_FC (−1)) than sensitive cases. Resilient cases also have a 5.879 thousand dollars higher square of effective rainfall (ER_NC_S) and 2.473 billion dollars higher square of average cash income level (ACIL_FC_S) than the sensitive cases.

The logistic regression was executed to further determine whether or not 36 capital indicators, e.g., 12 capital indicators themselves, their first-order lags and their squares, would predict the resilience of wheat to climate change. In total, in each model, among 12, 24, and 36 dependent variables, we assessed those with just two, three, or four significant influences on vulnerability, respectively. The outcome of five models indicated that ER_NC, ER_NC_S, ACIL_FC, ACIL_FC_S, ACIL_FC (−1), FSFI_SC, FSFI_SC_S, TCGR_NC_S, and FE_NC_S would reduce wheat climatic vulnerability significantly (see Table 4). Model 2, which attempted to indicate show the lag effect of capital on vulnerability, has fitted poorly since the significance of its Chi-square is smaller than 0.05. Many other variables in each model did not show significant statistical results, which indicates that the limited effects of livelihood capital on vulnerability.

**Table 4:** Logistic regression predicting resilience based on the capital indicator itself, its first-order lag and its square.

Models	Variables	B	S.E.	Wals	df	Sig.	Exp (B)	Cook	SR^2^	N	R^2^	OPC	test (Sig.)
1	ER_NC	0.017	0.006	6.846	1	0.009	1.017	<0.06	<2.40	91	0.475	78	6.991(0.538)
	ACIL_FC	0.000	0.000	14.057	1	0.000	1.000						
	FSFI_SC	0.000	0.000	11.208	1	0.001	1.000						
	C	−7.100	1.763	16.212	1	0.000	0.001						
2	ACIL_FC(−1)	0.000	0.000	18.841	1	0.000	1.000	<0.025	<1.75	85	0.460	71	14.198(0.048)
	C	−6.592	1.522	18.761	1	0.000	0.001						
3	TCGR_NC _S	0.000	0.000	4.944	1	0.026	1.000	<0.040	<2.30	90	0.592	83.3	4.910(0.767)
	ER_NC _S	0.000	0.000	7.145	1	0.008	1.000						
	ACIL_FC_S	0.000	0.000	17.801	1	0.000	1.000						
	FSFI_SC_S	0.000	0.000	3.815	1	0.051	1.000						
	C	−4.958	1.087	20.816	1	0.000	0.007						
4	ER_NC	0.015	0.007	3.885	1	0.049	1.015	<0.050	<2.10	73	0.653	80.8	5.017(0.756)
	FSFI_SC	0.000	0.000	10.954	1	0.001	1.000						
	ACIL_FC(−1)	0.000	0.000	13.239	1	0.000	1.000						
	C	−8.490	2.260	14.107	1	0.000	0.000						
5	ER_NC	0.056	0.021	7.213	1	0.007	1.058	<0.060	<2.50	81	0.846	93.8	0.53(1.000)
	ACIL_FC	0.000	0.000	11.233	1	0.001	1.000						
	FSFI_SC	0.000	0.000	10.299	1	0.001	1.000						
	FE_NC _S	0.000	0.000	4.924	1	0.026	1.000						
	C	−20.269	6.220	10.618	1	0.001	0.000						
6	FSFI_SC	0.000	0.000	11.703	1	0.001	1.000	<0.050	<2.40	71	0.664	83.1	9.975(0.267)
	ACIL_FC(−1)	0.000	0.000	12.482	1	0.000	1.000						
	C	−5.215	1.701	9.401	1	0.002	0.005						

Notes: C, Constant; SR^2^, Studentized residuals squares; R^2^, Nagelkerke R square; OPC, Overall percentage correct; Cook and SR^2^ is the range of selected samples after elimination of abnormal values.

Method: Forward: Conditional.

## Discussion

### Special assessments of wheat climatic vulnerability under the sustainable livelihood framework

A series of measurements of vulnerability have been used in climate change research under the IPCC framework. Crop-drought vulnerability is the ratio of the crop failure index (sensitivity, S) to the drought index (exposure, E) (*V = S/E*) ([10]. Agricultural vulnerability under climate change is the ratio of sensitive yield (S) to the product of adaptive yield (adaptive capacity, AC) and exposure degree (E) as follows: V = S/(AC*E) [51]. Wheat-drought vulnerability is presented as a function of the ratio of the product of exposure and sensitivity to the adaptive capacity (V = f(E*S)/AC) [52].

Unlike above-mentioned calculations of vulnerability, we indirectly assess vulnerability by comparing exposure and sensitivity. We draw on similar conclusions regarding Australian wheat climatic vulnerability from some previous studies [53, 54], which recommended increasing adaptive capacity without testing whether livelihood capital reduces vulnerability. For example, the index of adaptive capacity showed that South Australia and West Australia are relatively resilient at the state level [14]. This finding suggests that the classification of vulnerability through comparison of the *CI* with the *WFI* constitutes an effective means of expressing low and high vulnerability of wheat to climate change (responding to the resilient and sensitive groups). Additionally, the sensitive cases are seldom constrained by climate extreme events and the resilient cases are seldom supported by good wheat yield, which supports the finding of Gbetibouo, Ringler and Hassan (19) that regions with the most exposure to climate change are separate from the regions with high vulnerability or low adaptive capacity.

### Relations of the significant capital indicators to the climatic vulnerability of wheat

Our results showed that three NC indicators, one FC indicator, and one SC indicator are significantly related to wheat climatic vulnerability.

Three NCs are significant influences of vulnerability: effective rain (ER_NC) in Models 1 and 4 and its square in Model 3, the square of total crop gross revenues (TCGR_NC_S) in Model 3, and the square of fertilizer expenditures (FE_NC_S) in Model 5. The ER_NC can maintain ecological functions and provide a high adaptive capacity of wheat to climate change [55]. Moreover, the farmers in wheat sheep production zones cope with drought through harvesting rain [56] to reduce vulnerability. The ER_NC_S reflects the supply of effective rain that progressively decreases wheat climatic vulnerability. The TCGR_NC includes the main revenue from wheat, barley, oats and other crops, which reflects the complementation or substitutions between wheat and other crops. Thus, the TCGR_NC_S indicates the supply of crops that have a progressive increased resilience to climate changes. If wheat fails because of climate change, a high TCGR_NC_S means that the revenue may make up with the loss of wheat failure. The FE_NC acts on the wheat production through yield growth to reduce the climatic vulnerability [57], but usage of a lot of fertilizer induces groundwater salinization and contamination by nitrates, which enhances vulnerability to more severe climate change [58]. The FE_NC_S suggests that FE_NC progressively increases with the climatic resilience of wheat.

As hypothesized, higher average cash income level (ACIL_FC) in Model 1 and 5, its lag (ACIL_FC (-1)) in Model 4 and 6, and square (ACIL_FC_S) in Model 3 occur in the resilient cases. The ACIL_FC is helpful for the use and supply of irrigation, changing planting date, agro-forestry, and diversification of crop varieties [59, 60] to add adaptations and reduce vulnerability. This is then followed by the generation more income, increased welfare and improved food security in the achievements of livelihood outcomes [11] (Fig 1). The ACIL_FC progressively decreases with the climatic vulnerability of wheat.

Family share of farm income (FSFI_SC) in all significant models, as an SC indicator, includes at least four pathways to transforming adaptations to affect vulnerability both indirectly and directly. According to the four realms of SC including four different adaptations [61], FSFI_SC has four possible routes to reducing the climatic vulnerability of wheat. First, families collectively invest in farm infrastructure and raise tolerant-drought wheat. Second, families learn about climate information and adaptive technologies. Third, families activate latent social connections to obtain more assistance from friends and relatives. Fourth, families attend decision-making sessions in local networks to obtain additional help from communities.

Our retesting of the role of capital in the assessment of vulnerability makes our significant capital metrics different from capital indicators used in the extant research [14]. The reasons for such difference are as follows. First, we used different vulnerability metrics and various capital indicators because of the availability of data. Secondly, we tested the influence of capital on the vulnerability measured by the classification of resilient and sensitive groups, through logistic models for resilient and sensitive cases.

### Reasons for few capital indicators affecting vulnerability

We found that few significant capital indicators (e.g., three of 12 in Model 1, four of 24 in Model 5, two of 36 in Model 6) were related to vulnerability, which is similar to previous report that six of the 24 capital indicators were significantly related to adaptive capacity [62]. However, through comparing our construct model with the original SLF, we identified different reasons than previously reported. In Fig 1, besides the outcome of reducing vulnerability, the SLF have another livelihood outcomes, emphasizing on human perceptions to the vulnerability contexts, the portfolios of livelihood strategies, transformations and dynamical process and the order of proposed livelihood outcomes [2]. However, we focused on the role of a single capital indicator in the reduction of vulnerability, and ignored the other four keys of SLF (e.g., five-capital pentagon, structure and process, cognitive factors and the achieved order of livelihood outcomes) in Fig 1.

Firstly, the dotted five-capital pentagon (Fig 1) shows that we did not consider the asset connections or capital portfolios, e.g., the interactions between capital types and between capital indicators because of their complex and unavailability.

Secondly, the dotted triangles of structure and process (Fig 1) suggest that the influences of capital indicators on the vulnerability are uncertain under the interactions of these environmental influences. The SLF emphasizes the transforming structures of governments and private sectors, and the operational process of markets, laws, cultures, institutions, and policies. However, we were forced to ignore these dynamical transformations because they are too complicated to measure. We should disregard preconditions of implementing livelihood strategies without considering such correlated contexts in the selections of capital indicators.

Thirdly, we ignored cognitive factors, e.g., perceived vulnerability, is also a possible reason that most indicators of livelihood capital failed to reduce vulnerability [63].

Fourthly, we overlooked the achieved order of livelihood outcomes. Any livelihood outcomes are the integrated consequences of the portfolios of capital indicators and the transforming structures and processes. However, the farmers who implement these livelihood outcomes initially gained more income to fight poverty and hunger, increased their well-being, and gradually improved their food security. The reduced vulnerability is the fourth goal. The dotted square within the square of livelihood outcomes shows that we only focus on reduced vulnerability but ignore other aims and their achieving order.

Finally, several other limits from the data and measurements may obscure the role of capital indicators on reduced vulnerability. For example, the APSIM modeling only estimated the yield under constant management contexts (e.g. the same sowing date and fertilization time) for the different regions and seasons [64]. Furthermore, we excluded some invariant-time variables, such as soil moisture and land type [65].

## Conclusions

The purpose of this study was to determine the role of livelihood capital in the assessments and reductions of climatic vulnerability. We calculated a vulnerability index and classified resilient and sensitive cases of wheat to climate change for the Australian wheat—sheep production zone over the period from 1990 to 2010 to test the hypothesis (based on the SLF) that increasing livelihood capital reduces vulnerability. We also constructed a set of measures of regional adaptive capacity based on livelihood capital that includes financial, human, natural, physical, and social capitals. By testing for statistical differences between capital indicators for sensitive and resilient groups, we identified empirical correlations between wheat vulnerability to climate change and the 12 capital indicators. Notably, we could only verify 10 of 36 capital indicators that affect vulnerability. Furthermore, a serial of logistic models for resilient and sensitive cases are used to assess the impacts of each capital indicator, its first-order lag and the square of each capital indicator sampled on vulnerability. Similarly, two or four significant indicators are identified from 36 or 24 indicators, which again challenged the hypothesis that livelihood capitals effectively reduce vulnerability.

In this study, we advanced the existing understanding of the role of the increasing-capital method in the adaptations and concluded that further empirical reexaminations are required to test the relationships between capital measures and vulnerability under the SLF. The hypothesis that increasing livelihood capital can reduce vulnerability is supported by few capital indicators being related to vulnerability. While we concur that the SLF is a useful construct, we believe that significant work is required to make its operation useful. The historical memory and self-learning of farmers affects their resilience and future adaptation options in the assessment of vulnerability to climate change [66]. Therefore, to resolve these limitations, scholars should combine the SLF with other frameworks, e.g., the ecosystem services framework, diffusion theory, social learning, adaptive management, and transitions management [67]. This future research should focus on assessing the human perceptions of vulnerability, further capital portfolios, the order of livelihood outcomes, and integrating SLF with other frameworks.

## Supporting Information

S1 Dataset Capital indicator, wheat yield and temperature data. (XLSX)
